The article "Comparison of Montreal Cognitive Assessment in Korean Version for Predicting Mild Cognitive Assessment in 65-Year and Over Individuals" was published in 2022. Journal: Occup Ther Int.

# Comparison of Montreal Cognitive Assessment in Korean Version for Predicting Mild Cognitive Assessment in 65-Year and Over Individuals

**DOI:** 10.1155/2022/4108434

**Published:** 2022-04-19

**Authors:** Chiang-Soon Song, Hye-Sun Lee, Byung-Yoon Chun

**Affiliations:** ^1^Department of Occupational Therapy, College of Natural Science and Public Health and Safety, Chosun University, Republic of Korea; ^2^Department of Occupational Therapy, Kwangju Women's University, Republic of Korea; ^3^Department of Tax & Management, Gwangju University, Republic of Korea

## Abstract

**Objectives:**

The purpose of this study was to compare the validity and reliability of the two Korean versions of the MoCA for individuals aged ≥65 years.

**Methods:**

A total of 185 participants aged ≥65 years were included in this cross-sectional study. This study investigated the reliability of the two Korean versions of the MoCA (the MoCA-K and MoCA-K2) by having each participant complete both assessments twice and comparing them to their Korean version of the Mini-Mental State Exam (MMSE-K) scores. The participants either completed the tests in order A (MoCA-K2 before MoCA-K) then B (MoCA-K before MoCA-K2) or vice versa. The tests were then completed in the opposite order. This study conducted all experiments at 3-day intervals.

**Results:**

Of the 185 total participants analyzed, 95 indicated cognitive impairment, while 90 had normal in MoCA-K scores; 50 demonstrated cognitive impairment, while 135 had normal in MMSE-K scores; and 101 and 84 participants showed cognitive impairment and normal in MoCA-K2 scores, respectively. Cronbach's *α* values were 0.929 for the MoCA-K, 0.774 for the MMSE-K, and 0.919 for the MoCA-K2. The mean scores were 22.37, 25.29, and 21.96 points for the MoCA-K, MMSE-K, and MoCA-K2, respectively. The sensitivity and the specificity of the MoCA-K were 77.0% and 78.0%, respectively, while those of the MoCA-K2 were 68.9% and 80.0%, respectively.

**Conclusions:**

These results suggest that both the MoCA-K and MoCA-K2 are suitable and reliable evaluation tools for MCI screening; however, the MoCA-K had better overall sensitivity and specificity.

## 1. Introduction

In 2018, over 8.92% of the world's population was aged ≥65 years according to the Organization for Economic Cooperation and Development Labor Force Statistics [1]. The elderly Korean aged 65 and over accounted for 16.5% of the total population in 2021. Alzheimer's disease was the fifth leading cause of death among Korean people aged 65 and over in 2020 [2]. Mild cognitive impairment affects 36% of people aged ≥65 years in China, around 50% of whom will develop dementia within 3 years [3]. The decreased cognitive function involves impairments in memory, judgment, language, and attention caused by neurodegenerative or vascular deficiencies or dysthymia/dysphoria [4, 5]. Cognitive impairment can affect daily, functional, and social activities, ultimately resulting in poor quality of life [4, 6].

The article "Comparison of Montreal Cognitive Assessment in Korean Version for Predicting Mild Cognitive Assessment in 65-Year and Over Individuals" was published in 2022. Journal: Occup Ther Int.

Mild cognitive impairment (MCI) is a neurological disorder involving cognitive impairments greater than those expected from normal aging and education [4, 7–10]. MCI includes both memory and nonmemory impairments and may occur as a transitional stage between the normal aging-related cognitive decline and early dementia [8]. Therefore, MCI is not significant enough to interfere with instrumental activities of daily living and independent functioning. The cause of MCI remains unclear, although some of the possible risk factors are age, endocrine or cardiovascular dysfunction, vision and hearing loss, lower physical activity, and educational level, among others [4, 7, 8, 10]. To prevent progressive worsening and to treat MCI early, diagnostic tests and markers such as neuropsychological tests, neuroimaging, and biological markers should be incorporated into practice [8]. However, it is difficult to diagnose MCI due to the lack of sensitive and specific measurement tools, especially regarding memory loss.

The Montreal Cognitive Assessment (MoCA), which was developed in 1996 by Ziad Nasreddine, is a widely used screening tool for detecting MCI and has been validated in the clinical setting in patients with MCI [11]. This tool is meant to assess eleven different cognitive domains: attention and concentration, executive functions, memory, language, visuoconstructional skills, conceptual thinking, calculations, and orientation. The time required to administer the MoCA is approximately 10 minutes [11]. The total possible score is 30 points, and a score of 26 or more is considered normal. In 2017, the MoCA was available in a total of 46 languages [12–14].

Clinical measurement tools in English should be adapted in other countries based on linguistic and cultural translations [15]. Multiple cultural and linguistic variables may affect the norms of the MoCA across different countries and languages. There are two Korean versions of the MoCA, the MoCA-K and the MoCA-K2 [15, 16]. There are small differences in the items and score calculations between the two Korean versions of the MoCA [15, 16]. Therefore, different cut-off scores have been suggested for the two Korean versions of the scale to compensate for the education level of the population, and several modifications have been necessary to accommodate certain linguistic and cultural differences [15, 16]. However, neither version has been sufficiently validated, and it is not clear which of the two Korean versions is more reliable. Before using these tools in the clinical setting, it is essential that their validity and reliability be assessed sufficiently. Therefore, the purpose of this study was to compare the validity and reliability of the two Korean versions of the MoCA for individuals aged ≥65 years.

The article "Comparison of Montreal Cognitive Assessment in Korean Version for Predicting Mild Cognitive Assessment in 65-Year and Over Individuals" was published in 2022. Journal: Occup Ther Int.

## 2. Materials and Methods

### 2.1. Study Design and Data Collection

This study was a cross-sectional study of the two Korean versions of the MoCA (MoCA-K and MoCA-K2). All study participants provided written informed consent before the commencement of the study. G^∗^Power analysis was conducted to calculate the sample size before the primary outcome measures were performed. This study was measured by two occupational therapists and one physical therapist. To examine test-retest reliability, this study included four different scores per participant. The participants either completed the tests in order A (MoCA-K2 before MoCA-K) then B (MoCA-K before MoCA-K2) or vice versa. The tests were then completed in the opposite order. All experiments were conducted at 3-day intervals (Figure 1).

A total of 185 individuals who were aged ≥65 years participated in this study between December 7, 2020, and January 9, 2021. The participants had a sufficient understanding of the purpose and methodology of this study and participated voluntarily. The inclusion criteria were the following: (1) aged ≥65 years, (2) no diagnosed psychological diseases, (3) no visual field deficits, (3) no physical impairments, and (4) voluntary participation. Those who had participated in similar experiments in the previous 6 months, those who had depression, and those who were taking any medication which would affect the results of the experiments (such as antidepressants) were excluded from this study. All participants who dropped out before completing the study were also excluded. The study protocol was approved by the Kwangju Women's University Institutional Review Board (Permit No. 1041485-202009-HR-001-38) and conducted in accordance with the Declaration of Helsinki.

### 2.2. Measurement Tools

The primary measurements of this study were the MoCA-K and MoCA-K2 scores. The MoCA-K was adopted in 2008 by Lee based on the original MoCA version 7.1 (in English), which was designed as a rapid screening instrument for mild cognitive dysfunction and was used to evaluate different cognitive domains: (1) attention and concentration, (2) executive functions, (3) memory, (4) language, (5) visuoconstructional skills, (6) conceptual thinking, (7) calculations, and (8) orientation. The time required to administer the MoCA-K is approximately 10 minutes [13, 16, 17]. The total possible score is 30 points, and a score of 23 or above is considered to represent a normal cognitive function. The MoCA-K is not recommended if the participants are not able to reliably read and write. One point is added if the participant has ≥6 years of education. There are two main differences from the original version [13, 16]. First, the verbal fluency item in the MoCA-K requires the participant to list items that could be bought in the market, while the original version requires the participant to list as many words starting with letter F as possible in one minute. For both versions, a perfect score is given if the participant can say 11 words or more. Second, the two Korean versions of the MoCA give additional points depending on the years of education. The MoCA-K is based on ≥6 years of education, and the original is based on ≥12 years of education (Table 1) [13, 16].

The article "Comparison of Montreal Cognitive Assessment in Korean Version for Predicting Mild Cognitive Assessment in 65-Year and Over Individuals" was published in 2022. Journal: Occup Ther Int.

Kang et al. adopted the MoCA-K2 in 2009 based on the original MoCA version 7.1 (English) [15]. The MoCA-K2 was reported to have good reliability (Cronbach's *α* = 0.84, test-retest reliability intraclass correlation coefficient = 0.85) and validity (*γ* = 0.79) in a sample of normal older adult Korean participants (10). The tool includes items to assess visuospatial and executive function (5 points), naming (3 points), memory (5 points), attention (6 points), abstraction (2 points), language (3 points), and orientation (6 points) (Table 1) [15, 18].

The MMSE-K, a well-structured questionnaire to measure cognitive function, was translated into Korean and standardized by Kwon and Park in 1975 [19]. It consists of 12 items with 7 characteristics including orientation, memory registration, attention and calculation, recall, language, understanding and judgement repeat, and visual construction. It can be performed in a short time within 10 minutes and has little practice effect, so it has the advantage of being able to see changes over time by repeating measurements during the progression of disease [19]. Total scores of MMSE-K range from 0 to 30, and a score of ≥24 can be interpreted as normal cognitive function. The MMSE-K has previously been reported good validity for use in older adults [20].

### 2.3. Statistical Analysis

This study used descriptive statistics to analyze the demographic information of the participant. Cronbach's *α* was used to analyze the reliability of the three clinical tools, which included the MoCA-K, MMSE-K, and the MoCA-K2. A one-way ANOVA was used to analyze the differences between the three clinical tools, and the scheffe was used as a post hoc test to highlight exactly where these differences occurred. To analyze the sensitivity and specificity of the MoCA-K and the MoCA-K2, the receiver operating characteristic (ROC) curve was used in this study, and the selection criteria were applied by judging cognitive impairment based on the MMSE-K. The SPSS version 25.0 (IBM Inc., NY, USA) was used for all the statistical analyses. A *p* value < 0.05 was considered statistically significant.

The article "Comparison of Montreal Cognitive Assessment in Korean Version for Predicting Mild Cognitive Assessment in 65-Year and Over Individuals" was published in 2022. Journal: Occup Ther Int.

## 3. Results

### 3.1. Demographics of the Participants

Table 2 shows the demographics of the participants in this study. Sixty-three of the participants were male, and 122 were female. Additionally, 157 were diagnosed with various diseases, 154 of which were taking medications (42 for diabetes, 94 for hypertension, 24 for hyperlipidemia, 17 for osteoporosis, 3 for stroke, 5 for heart disease, and 36 for other reasons). 17 and 48 of the participants were smokers and daily drinkers, respectively.

The participants' cognitive dysfunction was examined using the MoCA-K, MMSE-K, and MoCA-K2 and determined according to the norm, a comprehensive neuropsychological evaluation tool. Of the 185 participants analyzed, 95 had MoCA-K scores in the cognitive impairment range, and 90 people had scores in the normal range. For the MMSE-K, 50 people showed cognitive impairment scores and 135 people had normal scores, and for the MoCA-K2, 101 people demonstrated cognitive impairment scores and 84 had normal scores (Table 2).

### 3.2. Reliability of the Three Clinical Tools

Table 3 shows Cronbach's *α* for the MoCA-K, MMSE-K, and MoCA-K2. The value was the strongest for the MoCA-K and the weakest for the MMSE-K. The values were 0.929 for the MoCA-K, 0.774 for the MMSE-K, and 0.919 for the MoCA-K2.

### 3.3. Comparison of the MoCA-K, MMSE-K, and MoCA-K2 Scores

This study analyzed the scores of the MoCA-K, MMSE-K, and MoCA-K2. The mean scores of the three clinical measurement tools were 22.37, 25.29, and 21.96 points, respectively. The differences in the scores between the three clinical measurement tools were statistically significant, with the highest being the MMSE-K score and the lowest being the MoCA-K2 score (Table 4).

To determine the presence of cognitive impairment, a cut-off score of 24 points or above was used for the MMSE-K. Since this is a comprehensive and widely used evaluation tool, this cut-off value was assumed to be correct. The sensitivity and the specificity of the MoCA-K were 77.0% and 78.0%, respectively, while those of the MoCA-K2 were 68.9% and 80.0%, respectively (Figure 2).

## 4. Discussion

The purpose of this study was to compare the validity and reliability of the two Korean versions of the MoCA for individuals aged ≥65 years. The main results of this study were the following: (1) the reliability of the three clinical tools was the highest for the MoCA-K and the lowest for the MMSE-K; however, while the MoCA-K and the MoCA-K2 had excellent reliability, the MMSE-K did not; (2) there were significant differences in the scores of the three evaluation tools; (3) assuming that the cut-off value for the MMSE-K was accurate, the sensitivity was higher with the MoCA-K and the specificity was higher with MoCA-K2. However, while the MoCA-K had fair values for both sensitivity and specificity, the MoCA-K2 had a fair specificity but a poor sensitivity value.

The article "Comparison of Montreal Cognitive Assessment in Korean Version for Predicting Mild Cognitive Assessment in 65-Year and Over Individuals" was published in 2022. Journal: Occup Ther Int.

In general, it is apparent that translating a clinical measurement tool from English into the language of another country requires alterations to reflect the language and culture of that country [21, 22]. Several cut-off scores have been suggested across different languages to compensate for the education level of different populations [22]. The validation study of the MoCA test by Nasreddine in 2005 showed that the MoCA was a promising tool for detecting MCI and early Alzheimer's disease compared with the well-known MMSE [11]. Other previous studies have shown conflicting results regarding the specificity and sensitivity of the MMSE-K and MoCA [23–25]. The MMSE and MoCA both have been translated into Korean [11, 13, 19]. Since the Korean standardization study was conducted in 1989, many researchers have studied the MMSE to confirm its reliability and validity in the older adults and in those with central nervous system disorders [19, 26, 27]. Although there are two Korean versions of the MoCA, studies on the reliability and validity of the two versions as well as their sensitivity and specificity have been insufficient. The MoCA-K and MoCA-K2 have different methods of scoring verbal fluency, and the MoCA-K reflected the education level of the participant in the score, whereas MoCA-K2 was not. It is presumed that such differences between the two evaluation tools would affect reliability and validity. Therefore, this study attempted to confirm the reliability and validity of the two Korean versions of the MoCA.

In Korea, the MMSE-K is being widely used as the primary screening tool for dementia in local community projects [28]. However, it is a well-known fact that the MMSE was not originally developed to diagnose dementia [29]. On the other hand, the MoCA was developed as an evaluation tool that can sensitively screen for MCI [11, 30–32]. Many studies have been conducted to assess how well the MoCA, a simple mental state test developed to be widely used and with no specific target group, can accurately be used to screen for specific clinical disorders such as dementia, stroke, and traumatic brain injury [30–32]. In this study, both the Korean versions of the MoCA were evaluated in old adults aged ≥65 years. There were statistically significant differences in the results of the MoCA-K and MoCA-K2; however, both evaluation tools showed excellent internal consistency. Using the MMSE-K score as a screening criterion, the results for sensitivity and specificity were both fair for the MoCA-K, while only the specificity was fair for the MoCA-K2. However, this interpretation may not be completely reliable since the statistical processes in this study were performed on the premise that the MMSE-K score realistically discriminates cognitive impairment. However, it is true that the MMSE-K is the most widely used evaluation tool for screening for dementia. In this study, although we conducted the evaluation with an interval of 3 days between two assessments (MoCA-K and MoCA-K2), it should not be concluded that the 3 days of interval would be suitable for preventing the learning effect of the continuous assessment.

The article "Comparison of Montreal Cognitive Assessment in Korean Version for Predicting Mild Cognitive Assessment in 65-Year and Over Individuals" was published in 2022. Journal: Occup Ther Int.

## 5. Conclusions

In summary, the results of this study suggest that the MoCA-K and MoCA-K2 are suitable and reliable evaluation tools for the screening of MCI. However, both the sensitivity and specificity were only fair with the MoCA-K. It should be emphasized that the education level is taken into consideration for MoCA-K scoring. This study was conducted with older adults to investigate the reliability and validity of a tool to assess cognitive decline. Future studies need to confirm the reliability and validity of the tools when used to assess for various diseases that may be associated with mild cognitive impairment in addition to the older adults. This study did not assess test-retest reliability. In addition, this study did not investigate the diagnosis of mild dementia by clinical specialists. These points should be considered in future studies.

## Figures and Tables

**Figure 1:** Flow diagram of the study.

**Figure 2:** ROC curve for the MoCA-K and MoCA-K2.

**Table 1:** Different items among MoCA, MoCA-K2, and MoCA-K.

Domains	MoCA 7.1 original	MoCA-K	MoCA-K2
Naming	(i) Naming (3 points)	(i) Naming (3 points)	(i) Naming (3 points)
Language	(i) Sentence repetition (2 points) (ii) Verbal fluency (*N* ≥ 11 words) (1 point) (iii) Language is assessed using a three-item confrontation naming task with low-familiarity animals (lion, camel, and rhinoceros; 3 points) (iv) Repetition of two syntactically complex sentences (2 points) and the aforementioned fluency task	(i) Sentence repetition (2 points) (ii) Verbal fluency (*N* ≥ 11 words) (1 point)	(i) Sentence repetition (2 points) (ii) Verbal fluency (*N* ≥ 6 words) (1 point)
Delayed recall	(i) Delayed recall (5 points) (ii) The short-term memory recall task (5 points) involves two learning trials of five nouns and delayed recall after approximately five minutes	(i) Delayed recall (5 points)	(i) Delayed recall (5 points)
Others	(i) Add 1 point if ≤12 yr edu	(i) Add 1 point, if ≤6 yr edu	

The article "Comparison of Montreal Cognitive Assessment in Korean Version for Predicting Mild Cognitive Assessment in 65-Year and Over Individuals" was published in 2022. Journal: Occup Ther Int.

**Table 2:** Common characteristics of the participants (*N* = 185).

Variables	Mean ± SD/frequency (percent)
Sex (male/female)	63 (34.1)/122 (65.9)
Age (yrs)	74.6 ± 6.6
Present disease (yes/no)	157 (84.9)/28 (15.1)
Medication (yes/no)	154 (83.2)/31 (16.8)
Diabetes	42 (22.7)
Hypertension	94 (50.8)
Hyperlipidemia	24 (13.0)
Osteoporosis	17 (9.2)
Vitamin K antagonist	3 (1.6)
Heart disease	5 (2.7)
Others	36 (19.5)
Smoking (yes/no)	17 (9.2)/168 (90.8)
Daily drinking (yes/no)	48 (25.9)/137 (74.1)
MoCA-K (≤22/≥23)	95 (51.4)/90 (48.6)
MMSE (≤23/≥24)	50 (27.0)/135 (73.0)
MoCA-K2 (≤22/≥23)	101 (54.6)/84 (45.4)

**Table 3:** Reliability of the three clinical tools (*N* = 185).

Variables	Cronbach's alpha
MoCA-K	0.929
MMSE-K	0.774
MoCA-K2	0.919

**Table 4:** Comparison of three clinical measurement tools for the cognitive impairments (*N* = 185).

Variables	Mean ± SD			*F*	*p*	Post hoc
	MoCA-K^a^	MMSE-K^b^	MoCA-K2^c^			
Cognition	22.37 ± 5.07	25.29 ± 3.34	21.96 ± 5.08	-13.448	<0.001	*b* > *a* > *c*

## Data Availability

Data are available upon request through contacting Dr. Byung-Yoon Chun as the corresponding author (email: steve.chun1@gmail.com).
